RETRACTED

# Empirical Investigation for Predicting Depression from Different Machine Learning Based Voice Recognition Techniques

**DOI:** 10.1155/2022/6395860

**Published:** 2022-04-07

**Authors:** R. Punithavathi, M. Sharmila, T. Avudaiappan, I. Infant Raj, S. Kanchana, Samson Alemayehu Mamo

**Affiliations:** ^1^Department of Information Technology, M.Kumarasamy College of Engineering (Autonomous), Karur, TN, India; ^2^Computer Science and Engineering, K. Ramakrishnan College of Technology, Trichy 621112, India; ^3^Department of Computer Science and Engineering, K. Ramakrishnan College of Technology, Trichy 621112, India; ^4^Department of Software Systems, PSG College of Arts & Science, Coimbatore 641014, TN, India; ^5^Department of Electrical and Computer Engineering, Faculty of Electrical and Biomedical Engineering, Institute of Technology, Hawassa University, Hawassa, Ethiopia

## Abstract

Over the past few decades, the rate of diagnosing depression and mental illness among youths in both genders has been emerging as a challenging issue in the present society. Adequate numbers of cases that have been prevailing had unheard of symptoms linked to mental depression that are able to be detected using their voice recordings and their messages in social media websites. Due to the wide spread usage of mobile phones, services and social sites emotion prediction and analyzing have been an indispensable part of providing vital care for the eminence of youth's life. In addition to dynamicity and popularity of mobile applications and services, it is really a challenge to provide an emotion prediction system that can collect, analyze, and process emotional communications in real time and as well as in a highly accurate manner with minimal computation time. Few depression prediction researchers have analyzed and examined that various social networking sites and its activities may be merged to low self-confidence, particularly in young people and adolescents. Moreover, the researchers suggest that several objective voice acoustic measures affected by depression can be detected reliably over the smart phones. And also in some observational study, it is stated that speech samples of patients from the telephone were obtained each week using an IVR system, and voice recording files from smart phones have been under process for predicting the depression. Such that several telephonic standards for obtaining voice data were identified as a crucial factor influencing the reliability and eminence of speech data. Hence, this article investigates on different process applied in different machine learning algorithms in recognizing voice signals which in turn will be used for scrutinizing the techniques for detecting depression levels in future. This will make a blooming change in the youth's life and solve the social unethical issues in hand.

RETRACTED

## 1. Introduction

One of the brainstorming issues in the recent medical field is the mental disorder due to depression occurring in the youths and adolescents of both genders. In the present contemporary world, Internet and its subsequent resources have become the nonstop sources of data with respect to an individual's opinion and emotions. Many Social media environments such as Face book, Twitter, and Whatsapp are one of the most frequent social circles where people regularly visit for collecting some information or suggestion, views, and outlook about several domains. Apart from the above, through voice call also people are sharing their emotions in many ways. Sentimental analysis and emotion analysis together tends to represent the privacy of the individual's mind state. In earlier times, there existed a number of emotion recognition systems through speech, video, image, or text. By analyzing the message in the SMS, one can easily detect the mindset of the user and once the mood is detected, the system can generate some type of “emoji” in order to indicate the emotion levels. By examining the video in perspective of detecting the stage of the emotion, a smart phone application will automatically be able to change the wallpaper or it will execute some media program files in favor of the user in order to deviate the mood. This type of process can also be applied to the voice conversation through the mobile phones in which the researchers apply the several machine learning algorithms for identifying the depression levels in their speech. A number of methods and algorithms have emerged in the modern speech technology system in which they depend on the interdisciplinary research area of signal processing and Artificial Intelligence. Machine Learning can be useful for building the right models using the right features to attain the right task. The new techniques evolved in machine learning paradigm have bought a huge process in the speech technologies. The major concept of machine learning is that learning from the given data set in order to analyze, detect, or conclude the task given. In addition to the above, various mathematicians, psychologist, engineers, medical researchers, computer scientists, and many others have invented and sometimes rediscovered several ways to solve the problems. Hence, in this comparative framework, the different techniques applicable for emotion prediction in voice recognition have been elaborated. This detailed statistical comparative analysis will shed light on the obtainable concepts on the research that in turn will pave the way for new innovations.

RETRACTED

## 2. Different Machine Learning Based Voice Recognition Techniques

The following sections will represent some diverse collections of Voice Recognition techniques based on Machine learning concepts. For every approach, its corresponding systematic process, working flow, and salient features are elucidated.

### 2.1. Articulatory-Based Speech Recognition

Articulatory phonology [1] is specifically based on the involvement of lip movements, tongue, and glottis, velum states in nature. By grouping all the parts in features, one can easily detect the states of asynchrony between the different streams among them. The pronunciation model was entirely based on the Articulator Features (AF), and every AF-based word [2] has been denoted by separate hidden streams with soft synchrony conditions applied. This in turn leads to the way for articulators such that they can move in a semi-independent way. These Soft synchrony conditions among the AF streams are formulated through asynchrony variables, where their distributions represent the probability of different number of states. An Asynchrony example illustrates that the state between lips or tongue and nasality produces the epenthetic stop fixing the vowel pronunciation. AF streams are also playing a vital role in the classifier-based observation modeling. Its applications have been involved in two approaches such as hybrid approach and tandem approach. In the hybrid approach, the hidden structure with the single stream of phonetic states is assumed. In this hybrid models, the Multilayer Perceptron (MLP) [2] outputs estimates the scaled likelihood format. Nondeterministic mapping from the phonetic state to AF state along with distribution states are used in this approach. The deterministic mapping between phones and AFs are already used in earlier AF-based hybrid model. This type of approaches produces cross domain and cross-lingual work in which the domain will have little data and attain low benefit from the classifiers on the data-rich domain activities such that these are language-independent components than the phones. In adherence with the tandem approach, MLP outputs are modeled with the Gaussian Mixture in the way of postprocessing, appending, and combining to the acoustic observation vector. Apart from that, this type of approach was also to be used in state-of-the-art large vocabulary systems. Hence, by observing various training data, the AF-based model drastically outperforms the standard phone-based monophonic model. Apart from the abovementioned factor, the articulatory features are also involved in the integrated part of automatic speech recognition. In this approach, the term of probabilistic lexical model is related between subword units in the lexicon pattern and the acoustic feature observation factored with the latent variables. The domain independent data [3] for acoustic system is highly trained along with phonemes and graphemes for producing efficiency in continuous speech recognition. The examination of the parameters of lexical model exemplifies that this approach adapts the knowledge-based phoneme to AF. In this automatic speech recognition system, the lexical units are statistically related to all acoustic units in nature. Let l^i^ be the lexical unit, and y^i^ be the D-dimensional probability vector, which in turn creates the probabilistic relationship between l^i^ and D-acoustic factors which is given in equation (1):

(1) yi=yil,…..yid,…..yiD^T,

where *y*_*i*_^*d*^=*P*(*a*^*d*^*|l*^*i*^) such that the above-stated lexical parameter has estimated the Kullback–Leibler divergence-based hidden Markov model (KL-HMM) approach in which it assumes the trained acoustic unit models. The pronunciation lexicon and word level transcriptions are used along with acoustic unit probability vector sequences. These parameters are used as a feature observation to train the HMM model in order to denote the lexical units. Every state is parameterized by a categorical value that gives the way for probabilistic relationship between acoustic and lexical units. Since feature observation and the state distributions are considered to be the probability vectors, KL divergence will compute the local scores at HMM states. In order to estimate the KL divergence, there are three possible ways generated such as.

RETRACTED

KL divergence (DKL)—In this case, the state distribution and reference distribution are the same:

(2) $$\begin{array}{c} D_{KL\;}\left(y_{i},z_{t}\right)=\overset{D}{\underset{d=1}{\sum }}y_{i}^{d}\log\left(\frac{y_{i}^{d}}{z_{t}^{d}}\right). \end{array}$$

Reverse KL divergence (DRKL)—In this case, the acoustic unit vector will be termed as the reference distribution:

(3) $$\begin{array}{c} D_{RKL\;}\left(y_{i},z_{t}\right)=\overset{D}{\underset{d=1}{\sum }}z_{t}^{d}\log\left(\frac{z_{t}^{d}}{y_{i}^{d}}\right). \end{array}$$

Symmetric KL divergence (DSKL)—In this case, the local score is the average of all local scores as *D*_*KL* _ and *D*_*RKL* _:

(4) $$\begin{array}{c} D_{SKL\;}\left(y_{i},z_{t}\right)=\;\frac{1}{2}\;\cdot \left[D_{KL\;}\left(y_{i},z_{t}\right)+D_{RKL\;}\left(z_{t},y_{i}\right)\right]. \end{array}$$

### 2.2. CNN-Based Continuous Speech Recognition

This Convolutional Neural Network (CNN) [4] is referred as the sequences of raw input signals, which are split into several frames and results in scores for each corresponding class. A temporal pooling layer and a nonlinearity layer combined with convolutional layer are involved in the filter process. After processing of the signal, the stages are fed into the classification stages, such that it will lead to multiple hidden layers. Apart from that it also gives the result as conditional probabilities *p*(*i|x*)) for each cluster *i* and for each frame *x*. Classical layers usually accept the fixed size input vectors, whereas convolution layer accepts the sequence of vectors and frames. A convolution layer [5, 6] performs well with the linear transformations for each and every successive window frames. Another kind of layer is called Max pooling layer in which it executes the local temporal max operations in aspect with input sequences. Hence, these types of layers gradually increase the robustness of the network to minor temporal distortions in the input sequences. In training the network, the parameters are learned by maximizing the log likelihood that can be given below as follows:

(5) $$\begin{array}{c} L\left(\theta \right)=\overset{N}{\underset{n=1}{\sum }}\text{log}\left(p\left(i_{n}|x_{n,}\theta \right)\right). \end{array}$$

By the way, the CNN-based system has the capability to perform the acoustic modeling process and feature learning paradigm from the raw input speech through the computation of posterior probabilities of context-dependent phonemes. For feature extraction or for matching the filters, the CNN-based model is acted upon. The systematic procedures [7] for these extraction initiates [8] with whole network training in the single database. After finalizing the weights of convolutional layer, the classification stage is executed to retrieve the desired result.

RETRACTED

### 2.3. Tandem-Based Speech Recognition

A tandem system [9] mainly deals with the multitraining data set for both Gaussian Mixture Model (GMM) training and neural network training. With the involvement of cross entropy and context-dependent targets, MLP has been trained by decision tree. The global semi-tied covariance matrix transforms the 26 dimensional bottleneck features and the HLDA project appends it with delta parameters. A fully designed tandem system will contain a speaker adaptive training system using global trained linear regression followed by Minimum Phone Error (MPE) [10] and Feature-spaced MPE (FMPE). Apart from this, a multipass decoding and adaption techniques are processed by using speaker independent decoding methods. Another tandem system named as SPINE 1 [10] has been framed to recognize the speech in an efficient manner and its working process was given below:

- Initially input raw speech is given into two feature extraction blocks.
- One feature block generates the Perceptual Linear Prediction (PLP) and the other calculates the Modulation filtered Spectrogram (MSG) features.
- By merging the above two feature blocks, the error reduction will be consequently reduced.
- The PLP feature contains the 13-element cepstrum in which everything is indulged with deltas and double deltas.
- The MSG consists of 14 spectral energy features which is split into two banks of modulation frequencies such as one is between 0 and 8 Hz and another is in the range of 8 and 16 Hz.
- After that, each feature system is fed up with its own neural network classifier.
- Each input acts as a window of successive features that provides temporal context.
- In this context, in order to enhance the symmetry and gaussianness of the distributions, neural network activations have been used.
- Finally, the sum of appropriate activations of two nets has been done to join the feature steams.
- Henceforth, it gives the most efficient performance in the small vocabulary works.

### 2.4. Hidden Markov Model (HMM)-Based Speech Recognition

The Hidden Markov Model (HMM) [11] is initially established for speech recognition in the form of discrete observation. The direct way of exploiting HMM was based on the vector quantization of feature extraction technique. In this, the sequence of speech signals will be converted to the collection of feature vectors that is extracted from the discrete distribution. The major advantage of the vector quantization from the complex signal processing is that few of the critical vector spaces are designed using sufficiently large codebook. The simple representation of codebook of vector quantization is projected in Figure 1.

Hierarchical clustering algorithms [12] are mainly used to construct the set of feature vectors for vector quantizer. Another two clustering techniques such as K-Means and LindeBuzo Gray algorithms are mainly used to reduce the dimensionality space by interchanging the group of words in the training database in order to represent the centroid range of points. In some cases of doing speech recognition with HMM, the Weighted Euclidean Measures are highly used for further accurate analysis. Thus, Vector quantization mainly used to map the feature vector to symbol and is also referred as the acoustic modeling system. This system represents the HMM state [13] and at the time of analysis, these symbols are matched against the unknown symbols, and finally it gives the way for detecting the voice nature and pitch of the input signal.

### 2.5. Deep Neural Network (DNN)-Based Large Vocabulary Continuous Speech Recognition

In this contemporary period, the Deep Neural Network (DNN) [14] has been achieving a tremendous endeavor for analyzing the Large Vocabulary Continuous Speech Recognition (LVCSR) process. These DNN in applying over the several datasets proved to be gaining results over the traditional Gaussian Mixture Model and Hidden Mixture Model approaches on a wide variety of small and large vocabulary continuous speech recognition. For reducing the Translation variance in the signals, the CNN will act as the alternate method of neural network to design the spatial and temporal correlation factors. Even though CNNs [6, 15] are more active and attractive where they are fully extensible and are used for the variety of acoustic models, but in some sort of processes, they capture translational invariance with far lesser parameters by duplicating weights across the time and frequency. Initially, the DNNs are not openly modeled for translation variance within voice signals where they exist for different styles of speech. Sometimes DNNs require a lot to apply large networks with many training samples. DNN also ignores the network topology without fully affecting the performance and optimization of the network. Hybrid DNN [7] is another technology for efficient use of speech recognition as it uses feature space speaker adapted (FSA) factors as input in a context of nine frames and as a current frame. All types of DNNs are fine trained prior through the cross entropy objective function proceeded by Hessian free sequence training. By using these DNN-based feature system, it is stated that 512 output targets has been trained. Apart from the above, by using DNN-based features [16, 17], GMM training is also applied to be at maximum likelihood. Thus, the above-stated way of processing also tends to be the most powerful method of speech recognition.

RETRACTED

### 2.6. Deep Recurrent Neural Network (DRNN)-Based Speech Recognition

Deep Recurrent Neural Networks [18] are powerful models that combine the multiple levels of presenting deep networks. It empowers the Recurrent Neural network (RNN) through flexible use of long-range context. In some cases, RNN efficiency [19] in speech recognition is very disappointing due to the output results obtained from the deep feed forward networks. At the initial stage, it attains the input sequence such as *x*=(*x*_1_,……, *x*_*T*_ ), where a standard RNN computes the hidden vector factors [20] such as follows: *h*=(*h*_1_,……, *h*_*T*_) and the output vector factors as *y*=(*y*_1_,……, *y*_*T*_), this in turn further iterates the equations from *t* = 1 to T. Deep RNNs are succeeding greatly by creating clusters of multiple RNN hidden layers [21] on top of each other of output sequences. Another technique called RNN transducers are also used for decoding the beam search to yield the good accuracy in acoustic raw input data.

### 2.7. Fuzzy Match-Based Syllable Level Speech Recognition

This Fuzzy match concept denotes the process of identifying the words and the sentences used as transcripts in the syllable sequence produced from speech recognition. Fuzzy match mainly determines the query word given by the user with the syllable string sequences in the transcript. The score obtained between the matching results tends to be the Levenshtein distance [22, 23] between the strings. Resulting distance value between the strings is weighted for each syllable word in the sequences. This method will easily reduce the common type of information miscommunication mistake done by the user in phoneme confusions. Final match will be confirmed with the document score containing highest syllable [24, 25] value that will act as the highest rank in finding the accuracy for recognition of nature of strings in the input. Additionally, Fuzzy logic also plays a vital role in differentiating the male and female speech in a given sample audio data. This variation process includes three different steps: fuzzification, generating fuzzy rules, and defuzzification. Initially in the fuzzification process, the system data is transformed to fuzzy data, and in that the triangular membership function is highly used to extract the fuzzy rules from the input audio data. The input data should be given to fuzzy logic [26] in the form of energy entropy, short time energy, and zero crossing rates such that the extracted output will be in the form of percentage of male and female speech signals.

## 3. Exploratory Analysis of Different Methods

Machine learning has been stated as one of the subdivision of Artificial Intelligence in which it has the higher capability of computing and learning from the prior experience data rather than explosively coded by the humans. This section specifically exemplifies the comparative analysis of the previously described different machine learning-based voice recognition methods based on the different attributes. The following Table 1 represents the machine learning approach names for speech recognition, dataset used for executing the algorithm, mathematical factors involved, dimensionality of the input used, accuracy gained in matching of the results, and their capabilities identified. The main thought of this contrast is not to investigate which is the best technique but to differentiate the approaches related to its behavioral performance, datasets used, and its salient features through which it highly gives the hand for the researchers to select the suitable recognition technique for prediction of depression levels in the youths as well as adulterants and thus it helps the medical diagnosis much better. Some of metrics that are used to evaluate the efficiency of each technique in their voice recognition is mentioned below.

RETRACTED

### 3.1. Word Error Rate (WER %)

The Word Error Rate (WER) is the most common performance metric that was frequently used to evaluate the efficiency of the voice recognition system. It mainly works at word level criteria, rather than the phoneme level. It is fully based on the power law, which states the correlation between the word error rate and the perplexity. This process initiates by aligning the spoken word sequence using the dynamic string alignment. It computes by adding up the source, insertions, deletions, and finally, it was divided by the total number of words in the reference.

### 3.2. Sentence Error Rate (SER%)

The Sentence Error Rate (SER) mainly indicates the percentage of sentences in which the translations have not been matched and contributes the sentence similarity measures in the speech data for recognition. If the given and resulted sentence mismatches, then it will detect the appropriate percentage.

### 3.3. Recognition Accuracy

The Recognition Accuracy is mainly dependent on some of the following factors:

- Increased error rates with the growing size of vocabulary
- Data size of confusable words
- Speaker dependence and independence
- Isolated or discontinuous or continuous
- Task and language constraints
- Acoustic signals
- Environmental noise in speech signal

## 4. Experimental Analysis of Different Methods

Thus all the above stated diverse collection of techniques has been experimented with the audio datasets in MATLAB R2013a in order to examine the quality and efficacy of the voice recognition approaches discussed.  Table 2 shows the results performed by the different machine learning-based voice recognition system and their corresponding Recognition Accuracy and Word Error Rates have been compared and analyzed.

The empirical outcomes of the voice recognition system on several audio datasets show that many of the techniques achieved highest accuracy rates over RM corpus data, Word Speaker system data, WSJ corpus data, and English broadcast news data. By the way, some algorithmic approaches need to be improved as regards their accuracy. In general, the higher accuracy rate techniques will be well suited for the prediction of the depression level in humans by recognizing their voice sounds in audio data. Finally, Figure 2 illustrates the pictorial analysis of each technique in their performance levels.

RETRACTED

In the below graph, the resulted values of accuracy, WER, and SER are examined based on the similarity measures, hence, it is identified that articulatory-based speech recognition, CNN, and DNN-based and also HMM-based speech recognition techniques perform well in their detection of voice data in a more accurate manner. Moreover, these mentioned machine learning methods if used for depression prediction, the researcher can easily predict the efficiency from its performance rates and can achieve the most optimized level in future medical diagnoses.

## 5. Review of Recent Few Depression Prediction Techniques through Feature Selection Methods

According to the World Health Organization (WHO), Depression and Anxiety disorders are the main route cause for several health issues. They have placed unwarranted burden on society, individuals, and families to a great extent. Some studies suggest that efficient and better treatments for depression can be easily handled by the earlier detection of the problems. Hence, in the following sections, some of the recent feature selection method of predicting depression in patient's audio data and their working methodologies has been elaborated.

### 5.1. Deep Convolutional Neural Network (DCNN)-Based Feature Extraction Method

Feature selection and Feature extraction [27] plays a vital role in predicting the severity of the depression levels. DCNN [28] supports the combination of hand-crafted features and spectral features for depression analysis. Low-level descriptors from the raw audio clips and Median Robust extended Local binary patterns features from the spectrograms of audio data set are extracted. After that process, DCNN is directly used for the analyzing the extracted data to learn the features. For an added advantage to the DCNN, the valuable characteristic information from the audiovisual signals is adopted. These deep learned features are selected based on the two deep network models. The first network model represents the audio features from the frame level waveforms, and the second network model represents the features from the spectrogram images.

For the extracted deep learned features, the frame level raw waveform has been fed into the first CNN [28] for learning filter bank representations. The resulted output features are mapped to the parameters of first CNN layer. The specific hyper parameters involved are filter length, number of filters, window size, Mel-size, and the number of Mel-bands. Finally, joint fine-tuning method is processed for boosting the performance of audio recognition. This method is also used in capturing the complementary information between the above said two network models. In this process, the Raw DCNN and the Spectrogram-DCNN are combined to detect the Beck Depression Inventory (BDI) scores separately. In the tuning process, four DCNN layers are created and joined as feature layers in both raw and spectrogram networks. And for regression process, Euclidean loss function is applied. Meanwhile, for reducing the risk of over fitting, dropout method is adopted. The extracted feature sets of DCNN are AVEC 2013 and GeMAPs.

RETRACTED

### 5.2. Affective Computing Methodology

Affective computing techniques [29] and methods are about the simulation of human affects and developments in the system of recognition. It can also be said as the interdisciplinary field of relating psychology and spanning computer science. This affective computing shows its vital roles in the depression detection and monitoring. In this computing, detection of depression is entirely based on the acoustic measures of voice and its extracted features. The most widely retrieved acoustic features of the dataset are as follows:

- Fundamental Frequency—This parameter approximates the average rates of glottis opening and closing in voice signals
- Formants—Peak frequency obtained from Fourier analysis.
- Power Spectral Density (PSD)—Strength of signal energy that acts as a function of frequency.
- Speaking Rate—Represents the number of words spoken per minute.
- Mel Frequency Cepstral Coefficients—These are the logarithmic coefficients correlated to the audio signals.

Hence, the knowledge extracted from the person's mood through affective computing methodologies will be send to the medical specialist for continuous follow-up and provide therapies for patients.

### 5.3. openSMILE Machine Learning Tool

This openSMILE tool[30] was mainly used in the feature extraction process from the collected acoustic signals. With these retrieved features, detection of depression is in ease of case. Some of them are listed below:

- Loudness
- Fundamental Frequency (F0)
- F0 Envelope
- Line Spectral Pairs (LPS)
- Zero Crossing Rate
- Voicing probability
- Mel frequency Cepstrum Coefficients

### 5.4. Ensemble-Based 1d-CNN Algorithm

Generally, ensemble methods are the meta-algorithms in which several machine learning techniques are combined to promote the prediction's efficiency and improvement in existing methodologies. In this approach, ensemble averaging method [31] is implemented to combine the sample outputs produced by different prediction algorithms. The audio files of each patient, which are associated with their PHQ-8 score are taken from the Distress Analysis Interview Corpus Wizard database. These files are preprocessed for better prediction analysis. In order to classify the audio recordings into depressed and nondepressed part, the PHQ-8 scores are processed into binary labels as 0 for nondepressed and 1 for depressed. In preprocessing stage, the second voice of the interviewers involved in each patient's audio file has been removed. All those processes are implemented using diarization algorithm embedded in *Python* library as “PyAudioAnalysis.” The speech features of the audio data are extracted with the help of Octave toolbox. This detection system is composed of two modules as CNN-based classification and aggregation of several predictions by means of Ensemble method for improving accuracy. In the first module process, a few sets of preliminary tests are done on some classical architectures as normal-like image analysis. Since the speech signals are of log spectrogram, while handling in the network, it will be considered as a whole image. These types of methods are considered as different squared network architectures. The obtained results are not completely satisfactory due to the spatial distribution of log spectrum pixels, in which it does not have the similar relationships.

RETRACTED

However, in order to overcome the above difficulties, one-dimensional CNN (1d-CNN) was implemented directly over the frequency axis instead of two-dimensional kernels. This new network methodology consists of one input layer, one output layer, and four intermediate layers. Hence, capturing the frequency correlations at the short-term level was done with the above configuration level. The depression prediction has been done with each speaker's input audio file. To promote more accurate results, averaging the probabilities of samples has been taken for ensemble process. Based on the availing results, final speaker label was identified for corresponding predicted depression level.

### 5.5. Machine Learning-Based Behavioral Diagnosis

In the field of psychiatry, diagnostic measures and its treatment tend to be a tedious task. To make the prediction quicker and simpler, behavioral machine learning methods [32] are contributing a lot for the specificity and sensitivity of the depression and anxiety diagnosis. Machine-based assessments always seem to be the better decision while comparing with the perspective of well-trained clinicians, and it helps in identifying the suitable treatments. Additionally, cognitive biases and machine learning based diagnosis [33] are playing a vital role in increasing the diagnostic sensitivity by allowing the detection of the differences in healthy and nonhealthy individuals from the data given. Despite these remarkable merits of machine learning approaches, still few diagnoses of certain researches are experiencing substantial difficulties. Hence, more innovative techniques are needed to aggregate findings and develop new approaches and methodologies that can be incorporated by mental health diagnoses and other clinicians and institutions.

RETRACTED

## 6. Conclusion

Depression level prediction among the youths and elderly persons are becoming one of vast and crucial situation in this contemporary society. It is gaining more and more needs and requirements from the medical diagnosis and researchers. In the process of emotion detection from the audio speech of social media and as well as voice call recordings of smart phones and machine learning algorithms are playing a vital role in attaining the accuracy levels in achieving the target goal. Consequently, this proportional and theoretical study of different collection of speech recognition explores its nature of working paradigm and its individuality in a specific keen manner. Herewith, the original contribution of this study is the methodological and systematic working flow of each technique in a statistical manner. Finally, the comparison table results, proves that still many algorithms need to be improved in order to achieve the optimality in accuracy levels. Hence, this examination of different techniques makes better understanding for the readers as well as for the medical researchers in analyzing and treating the mentally depressed persons in an effective manner as this comparative review article will make the machine learning researchers to innovate more techniques to solve the problems in hand.

### 6.1. Avenues for Future Enhancement

As further research, the future work will be focused on collaboration of Machine and Human science that will incorporate the prior predictions of Prenatal Mental Retardation disorders and thus it will be used for detecting the early signs of health issues to prevent baby syndrome.

## Figures and Tables

**Figure 1:** Vector quantization process.

**Figure 2:** Statistical analysis of performance metrics.

**Table 1:** Descriptive analysis of each technique.

Approach name	Algorithm/Mathematical factors involved	Performance highlights	Dataset name	Dimensionality of dataset
Articulatory-based speech recognition (ABSR)	Probabilistic lexical modeling and GMM components	Having high lexical access and used for multichannels	RM corpus and mono phone baseline	3.8 Hz of speech data
CNN-based continuous speech recognition (CNN-BSR)	Convolutional layer and max pooling layer	Generalization of large amount of data in efficient manner	WSJ corpus	SI-284 sets and 16 KHz with 80 hours of speech data
Tandem-based speech recognition (TBSR)	SPINE 1 tandem recognizer	Effectively used with high background noise audio data	MFC with delta and double data	8 hours of recordings data
HMM-based speech recognition (HMM-BSR)	Vector quantization method and clustering algorithms	Gives good resemblance between varying speech data	Word speaker independent system	1000 words speaker
DNN-based vocabulary speech recognition (DNN-BSR)	Convolutional and fully connected convolutional layer	Results in optimal level of attaining accuracy in fully connected layers	English broadcast news	400 hours audio
DRNN-based speech recognition (DRNN-BSR)	Recurrent neural network training system	It has high bidirectional short-term memory	TIMIT corpus data	462 speaker sets
Fuzzy match-based speech recognition (FBSR)	Fuzzy matching algorithmic process	More faster accessing of the syllable word sequences	145 broadcast news from BURSC corpus	7242 queries words audio

RETRACTED

**Table 2:** Comparison of Recognition Accuracy and WERs of Different approaches.

Approach name	Recognition accuracy	WER	SER
ABSR	0.956	0.044	0.10
CNN-BSR	0.901	0.099	0.87
TBSR	0.713	0.287	0.342
HMM-BSR	0.963	0.37	0.43
DNN-BSR	0.889	0.111	0.44
DRNN-BSR	0.763	0.237	0.445
FBSR	0.86	0.14	0.34

## Data Availability

The data used to support the findings of this study are included in the article. Should further data or information be required, these are available from the corresponding author upon request.

## References

[1] Aradilla G., Bourlard H., Magimai-Doss M. (2008). Using KL-based acoustic models in a large vocabulary recognition task. *Proceedings of Inter speech*.

[2] Aradilla G., Vepa J., Bourlard H. (2007). An acoustic model based on Kullback–Leibler divergence for posterior features. *Proceedings of ICASSP*.

[3] Abdel-Hamid O., Mohamed A.-r., Jiang H., Deng L., Penn G., Yu D. (2014). Convolutional neural networks for speech recognition. *IEEE/ACM Transactions on Audio, Speech, and Language Processing*.

[4] Jiang H. (2010). Discriminative training of HMMs for automatic speech recognition: a survey. *Computer Speech & Language*.

[5] Xiaodong He X., Li Deng L., Wu Chou W. (2008). Discriminative learning in sequential pattern recognition. *IEEE Signal Processing Magazine*.

[6] Seide F., Li G., Yu D. (2011). Conversational speech transcription using context-dependent deep neural networks. *Proceedings of the Interspeech*.

[7] Sainath T. N., Kingsbury B., Ramabhadran B., Fousek P., Novak P., Mohamed A. (2011). Making deep belief networks effective for large vocabulary continuous speech recognition. *IEEE Workshop Automation Speech Recognition*.

[8] Zhu Q., Chen B., Morgan N., Stolcke A. (2005). Tandem connectionist feature extraction for conversational speech recognition. *Machine Learning for Multimodal Interaction*.

RETRACTED

[9] Rasipuram R., Magimai-Doss M. (2015). *Articulatory Feature Based Continuous Speech Recognition Using Probabilistic Lexical Modeling*.

[10] Hermansky H., Ellis D. P., Sharma S. (2000). Tandem connectionist feature extraction for conventional HMM systems. *Speech, Signal Process*.

[11] Morgon N., Bourland H., Cohen M., Franco H. (1993). Hybrid neural network/hidden Markov model system for continuous speech recognition. *International Journal of Pattern Recognition and Artificial Intelligence*.

[12] Konig Y., Morgan N., Chandra C. (1991). *GDNN: A Gender-dependent Neural Network for Continuous Speech Recognition*.

[13] Murveit H., Cohen M., Price P., Baldwin G., Weintraub M., Berntein J. (February 1989). *DARPA Speech and Natural Language Workshop*.

[14] Levinson S. E., Rabiner L. R., Sondhi M. M. (1983). An introduction to the application of the theory of probabilistic functions of a Markov process to automatic speech recognition. *Bell System Technical Journal*.

[15] Dahl G. E., Dong Yu D., Li Deng L., Acero A. (2012). Context-dependent pre-trained deep neural networks for large-vocabulary speech recognition. *IEEE Transactions on Audio Speech and Language Processing*.

[16] Pan J., Liu C., Wang Z., Hu Y., Jiang H. (2012). Investigation of deep neural networks (DNN) for large vocabulary continuous speech recognition: why DNN surpasses GMMs in acoustic modeling. *Proceedings of the ISCSLP*.

[17] Hinton G., Deng L., Yu D. (2012). Deep neural networks for acoustic modeling in speech recognition: the shared views of four research groups. *IEEE Signal Processing Magazine*.

[18] Kingsbury B., Sainath T. N., Soltau H. (2012). Scalable Minimum bayes risk training of deep neural network acoustic models using distributed hessian-free optimization. *Proceedings of the Inter Speech*.

[19] Robinson A. J. (1994). An application of recurrent nets to phone probability estimation. *IEEE Transactions on Neural Networks*.

[20] Oriol Vinyals, Ravuri S., Povey D. Revisiting recurrent neural networks for robust ASR.

[21] Maas A., Le Q., O’Neil T., Vinyals O., Nguyen P., Ng A. (2012). *Recurrent Neural Networks for Noise Reduction in Robust Asr*.

[22] Meng H. M., Lo W. K., Li Y. C., Ching P. C. Multiscale audio indexing for Chinese spoken document retrieval.

[23] Chen B., Wang H., Lee L. (2002). Discriminating capabilities of syllable-based features and approaches of utilizing them for voice retrieval of speech information in Mandarin Chinese. *IEEE Transactions on Speech and Audio Processing*.

[24] Larson M., Eickeler S., Paass G., Leopold E., Kindermann J. (2002). Exploring sub word features and linear support vector machines for German spoken document classification. *Proceedings of ICSLP*.

RETRACTED

[25] Larson M., Eickeler S. Using syllable-based indexing features and language models to improve German spoken document retrieval.

[26] Ganapathiraju A., Hamaker J., Ordowski M., Doddington G., Picone J. (2001). Syllable-based large vocabulary continuous speech recognition. *IEEE Transactions on Speech and Audio Processing*.

[27] Yasin O., Merve D., cenk R. (2019). *Depression Screening from Voice Samples of Patients Affected by Parkinson’s Disease*.

[28] Lang He, Cui C. (2018). Automated Depression analysis using Convolutional neural network from speech. *Journal of Biomedical Informatics*.

[30] Wang J., LeiZhang T., Pan W., Hu B., Zhu T. (2019). Acoustic Differences between healthy and depressed people: a cross situation study. *BMC Psychiatry research article*.

[31] Vázquez-Romero A., Gallardo-Antolín A. (2020). Automatic detection of depression in speech using ensemble convolutional neural networks. *Entropy*.

[32] Richter T., Fishbain B., Levin G. R., Singer H. O. (2021). Machine learning based behavioral diagnostic tools for depression: advances, challenges and future directions. *Journal of Personalized Medicine MDPI*.

[33] Chung J., Teo J. (2022). Mental health prediction using machine learning: taxonomy, applications and challenges. *Hindawi Applied Computational Intelligence and Soft Computing*.

